# The Role of HOTAIR/miR-148b-3p/USF1 on Regulating the Permeability of BTB

**DOI:** 10.3389/fnmol.2017.00194

**Published:** 2017-06-28

**Authors:** Libo Sa, Yan Li, Lini Zhao, Yunhui Liu, Ping Wang, Libo Liu, Zhen Li, Jun Ma, Heng Cai, Yixue Xue

**Affiliations:** ^1^Department of Neurobiology, College of Basic Medicine, China Medical University Shenyang, China; ^2^Key Laboratory of Cell Biology, Ministry of Public Health of China, and Key Laboratory of Medical Cell Biology, Ministry of Education of China, China Medical University Shenyang, China; ^3^No. 1 English Department, School of Fundamental Sciences, China Medical University Shenyang, China; ^4^Department of Neurosurgery, Shengjing Hospital of China Medical University Shenyang, China; ^5^Liaoning Research Center for Translational Medicine in Nervous System Disease Shenyang, China

**Keywords:** blood tumor barrier, HOTAIR, miR-148b-3p, USF1, tight junction related proteins

## Abstract

Homeobox transcript antisense intergenic RNA (HOTAIR), as a long non-coding RNA (lncRNA), has been considered to play critical roles in the biological properties of various tumors. The purposes of this study were to investigate the role and possible molecular mechanisms of HOTAIR in regulating the permeability of blood tumor barrier (BTB) *in vitro*. Our present study elucidated that the expressions of HOTAIR and upstream stimulatory factor 1 (USF1) was up-regulated, but miR-148b-3p was down-regulated in glioma microvascular endothelial cells (GECs). Knockdown of HOTAIR could increase the permeability of BTB as well as down-regulated the expressions of tight junction related proteins ZO-1, occludin, claudin-5, but up-regulated miR-148b-3p expressions in GECs. Meanwhile, dual-luciferase reporter assays demonstrated that HOTAIR was a target RNA of miR-148b-3p. Furthermore, overexpression of miR-148b-3p increased the permeability of BTB by down-regulating the expressions of tight junction related proteins and USF1 in GECs, and vice versa. And further result revealed USF1 was a target of miR-148b-3p. Silence of USF1 increased the permeability of BTB duo to their interaction with the promoters of *ZO-1, occludin*, and *claudin-5* in GECs. Taken together, our finding indicated that knockdown of HOTAIR increased BTB permeability via binding to miR-148b-3p, which further reducing tight junction related proteins in GECs by targeting USF1. Thus, HOTAIR will attract more attention since it can serve as a potential target of drug delivery across BTB and may provide novel strategies for glioma treatment.

## Introduction

Malignant glioma has been overwhelmingly considered as the most common primary tumor in the brain (Li et al., 2014). Due to the presence of blood tumor barrier (BTB), macromolecular chemotherapeutic agents are arduous to reach the tumor tissues and dramatically attenuate the chemotherapeutic effect. Accordingly, selective BTB opening is an effective method to improve chemotherapeutic efficacy of brain glioma (Black and Ningaraj, 2004; Wang and Liu, 2009; Wang et al., 2015).

Long non-coding RNAs (lncRNAs) are one of RNA species with a length of more than 200 nucleotides, which don't participate in encoding proteins, but are involved in regulating gene expression on a wide scale, such as transcription or post-transcription regulation and epigenetics (Mercer et al., 2009; Zhou et al., 2016). Homeobox transcript antisense intergenic RNA (HOTAIR) is currently one of the most researched lncRNAs. Extensive research has revealed HOTAIR is closely related to the development and progression of various tumors. HOTAIR is highly expressed in breast cancer, lung cancer, pancreatic cancer, hepatocellular carcinoma, gastric cancer, brain glioma and related to metastasis and poor prognosis of tumor, which strongly indicating HOTAIR plays carcinogenic role in the above mentioned cancer tissues (Gupta et al., 2010; Geng et al., 2011; Hajjari et al., 2013; Kim et al., 2013; Zhang et al., 2013; Zhuang et al., 2013). It has been report that HOTAIR was involved in regulates malignant biological behaviors of glioma cells by targeting miR-148b-3p (Wang G. et al., 2016). However, there is no report about the role and mechanism of HOTAIR in regulating glioma microvascular endothelial cells (GECs) function and further modulating the permeability of BTB. Several studies suggested lncRNAs, as competing endogenous RNAs (ceRNAs), could bind to miRNAs and play pivotal roles in the process of post-transcription regulation (Salmena et al., 2011). For example, HOTAIR inhibited the regulatory role of miR-331-3p in HER2 expression of gastric cancer tissue (Liu et al., 2014). And HOTAIR can suppress the expression of miR-7, which inhibit SETDB1 expression to further influence the proliferation, invasion and metastasis of breast cancer stem cells (Zhang H. et al., 2014). Bian has reported that HOTAIR may act as an endogenous “sponge” of miR-148b, which regulates expression of the DNMT1/MEG3/p53 pathways in hepatic stellate cells (Bian et al., 2017). All the above studies inferred that HOTAIR might inhibit the expressions of miRNAs and result in the changes of downstream related molecules to further regulate the biological function of cancer cells.

MicroRNAs are small single strand non-coding RNAs consisting of 18–22 nucleotides and regulate gene expression through the interaction with 3′untranslated region (3′UTR) of target genes (Bartel, 2004). MiR-148b-3p is included in miR-148/152 family, which is differentially expressed in gastroenteric tumor and takes part in tumor growth, proliferation, apoptosis, angiogenesis drug susceptibility, and other biological functions (Chen et al., 2010). Recently studies found the expression of miR-148b-3p was up-regulated in lung adenocarcinoma cells, and influenced the response of lung adenocarcinoma cells to hypoxia through regulating NOG and WNT10B genes (Geng et al., 2016). And miR-148b-3p was also highly expressed in breast cancer and promoted the proliferation of breast cancer cells (Aure et al., 2013). However, it has been reported miR-148b-3p was down-regulated in gastric cancer cells and regulated various target genes to involve in the regulation of Wnt, MAPK, and Jak-STAT signaling pathways (Luo et al., 2015). Nevertheless, the expression of miR-148b-3p in GECs and whether miR-148b-3p is involved in regulating BTB permeability mediated by HOTAIR has not been reported until now.

Upstream stimulating factor (USF) includes upstream stimulating factor 1 (USF1) and upstream stimulating factor 2 (USF2), which belongs to the basic helix-loop-helix leucine zipper family of transcription factors. As an important regulatory factor, USF has highly conserved bHLH-LZ domain and binds to consensus sequence (CANNTG) of E-box to further regulate the transcription process of different proteins (Wu et al., 2013; Lupp et al., 2014). USF1 was reported to regulate the expression of IL-10 in glioma related microglia: inhibition of USF1 expression resulted in the up-regulation of IL-10 expression (Zhang et al., 2007). In liver cancer HepG2 cells, USF1 resisted oxygen sugar deprivation induced apoptosis by regulating miR-132 (Wang et al., 2014). However, whether USF1 is involved in regulating the function of GECs or the permeability of BTB and its possible mechanism still remained unclear.

The purposes of this study were to investigate the role and possible molecular mechanisms of HOTAIR in regulating the permeability of BTB *in vitro*. The present study firstly investigated the endogenous expressions of HOTAIR, miR-148b-3p, and USF1 in GECs, and secondly investigated the roles of HOTAIR, miR-148b-3p, and USF1 in the permeability of BTB, respectively, and further explored their potential mechanisms. It is aim to find new targets and methods for opening BTB selectively and improving chemotherapeutic efficacy.

## Materials and methods

### Cell lines and culture

The human cerebral microvascular endothelial cell line hCMEC/D3 marked as “ECs,” was kindly provided by Dr. Couraud (Institute Cochin, Paris, France). The cells were cultured in endothelial basal medium (EBM-2; Lonza, Walkersville, MD, USA), supplemented with 5% fetal bovine serum (FBS; PAA Laboratories GmbH, Pasching, Austria), 1.4 μmol/L hydrocortisone (Sigma-Aldrich, St. Louis, MO, USA), 1% chemically defined lipid concentrate (Life Technologies Corporation, Paisley, UK), 5 μg/ml ascorbic acid (Sigma-Aldrich, St. Louis, MO, USA), 1 ng/ml human basic fibroblast growth factor (bFGF; Sigma-Aldrich, St. Louis, MO, USA), 10 mM HEPES(PAA Laboratories GmbH, Pasching, Austria). Human glioblastoma U87 cell line and human embryonic kidney (HEK) 293 T cell line were purchased from the Shanghai Institutes for Biological Sciences Cell Resource Center (Shanghai, China). Both U87 and HEK 293 T cells were cultured in high glucose Dulbecco's modified Eagle's medium (DMEM) supplemented with 10% fetal bovine serum. All cells were maintained in a humidified incubator at 37°C with 5% CO_2_. The medium was renewed every 2 days.

### Establishment of BTB model *in vitro*

BTB model in vitro was established by co-culturing ECs and U87 cells with Transwell permeable support systems (0.4 μm pore size; Corning, NY, USA). U87 cells were seeded at 2 × 10^4^ per well into lower chamber of 6-well Transwell inserts with a suitable amount of DMEM till the cells were confluent. ECs were subsequently seeded at 2 × 10^5^ per well into upper chamber of 6-well Transwell inserts, coated with 150 μg/ml Cultrex Rat Collagen. The cells were co-cultured for 4 days with EBM-2 in both lower and upper chambers. The medium was then refreshed every 2 days. Thus, BTB model was established successfully and glioma microvascular endothelial cells marked as “GECs” were obtained. In the subsequent experiments, either un-transfected or transfected cells were GECs of BTB models in vitro, unless otherwise indicated (for example Figure 1).

**Figure 1:** The endogenous expressions of HOTAIR, miR-148b-3p, and USF1 in ECs and GECs. **(A,B)** Relative expressions of HOTAIR and miR-148b-3p in ECs and GECs were detected by qRT-PCR. **(C,D)** Relative protein expression of USF1 in ECs and GECs were detected by western blot. The IDVs were shown using GAPDH as an endogenous control. Data represent mean ± SD (**A**: *n* = 4; **B–D**: *n* = 3, each group). ^*^P < 0.05 and ^**^P < 0.01 vs. ECs group.

### Cell transfection and generation of stable cell lines

Knockdown of HOTAIR regulated the permeability of BTB, but not BBB *in vitro* in pre-experiment (Supplement Figure 1), thus we just focus on BTB in this study. The short hairpin RNA against human HOTAIR gene (shHOTAIR; sense: CACCGCCTTTGCTTCGTGCTGATTCTTCAAGAGAGAATCAGCACGAAGCAAAGGCTTTTTTG; antisense: GATCCAAAAAAGCCTTTGCTTCGTGCTGATTCTCTCTTGAAGAATCAGCACGAAGCAAAGGC) was constructed into pGPU6/GFP/Neo plasmid vector (GenePharma, Shanghai, China) which was transfected into cells and might lead to knockdown of HOTAIR [marked as “HOTAIR (−)”]. The plasmid carrying a non-targeting control sequence was used as a negative control (NC) of short hairpin HOTAIR. The experimental cells were divided into three groups: control (un-transfected) group, HOTAIR (−) NC group, and HOTAIR (−) group.

Human USF1 coding sequence (CDS) was ligated into the pIRES2-EGFP vector (GenScript, Piscataway, NJ, USA) to overexpress USF1 [marked as “USF1 (+)”]. Empty pIRES2-EGFP vector was used as NC of USF1 (+). Short hairpin directed against human USF1 gene (shUSF1; sense: CACCGCCAGAGTAAAGGTGGGATTCTTCAAGAGAGAATCCCACCTTTACTCTGGCTTTTTTG; antisense: GATCCAAAAAAGCCAGAGTAAAGGTGGGATTCTCTCTTGAAGAATCCCACCTTTACTCTGGC) was ligated into pGPU6/GFP/Neo vectors (GenePharma, Shanghai, China) to silence USF1 [marked as “USF1 (−)”]. Plasmid carrying a non-targeting sequence (sense: CACCGTTCTCCGAACGTGTCACGTCAAGAGATTACGTGACACGTTCGGAGAATTTTTTG; antisense: GATCCAAAAAATTCTCCGAACGTGTCACGTAATCTCTTGACGTGACACGTTCGGAGAAC) was used as a NC of USF1 (−). The experimental cells were divided into five groups: control group, USF1 (+) NC group, USF1 (+) group, USF1 (−) NC group, and USF1 (−) group.

Transfection was performed in 24-well plates when ECs at ~60–80% confluence by using Lipofectamine LTX and Plus Reagents (Life Technologies Corporation, Carlsbad, CA, USA) according to the manufacturer's instructions. After 48 h of transfection, the cells were subjected to G418 (Sigma-Aldrich, St. Louis, MO, USA). The stable transfected cells were selected by the culture medium containing 0.4 mg/ml G418. G418-resistant cell clones were established after about 3–4 weeks. The efficiencies of stable transfected HOTAIR cell lines were assessed by real-time PCR (Supplement Figure 2A). The efficiencies of stable transfected USF1 cell lines were verified by western blot analysis.

### Cell transfection of MicroRNA

The miR-148b-3p agomir (sequence: 5′-UCAGUGCAUCACAGAACUUUGU AAAGUUCUGUGAUGCACUGAUU-3′) or NC (sequence: 5′-ACAAAGUUCUGUGAUGCACUGA-3′), miR-148b-3p antagomir (sequence: 5′-UUCUCCGAACGUGUCACGUTTACGUGACACGUUCGGAGAATT-3′) or their NC (sequence: 5′-ACAAAGUUCUGUGAUGCACUGA-3′) were synthesized (GenePharma, Shanghai, China). ECs were transiently transfected using lipofectamine 3000 reagent (LifeTechnologies Corporation, Carlsbad, CA, USA) according to protocols. After 48 h, transiently transfected cells could be used in the subsequent experiments. The efficiencies of transfection were assessed by real-time PCR (Supplement Figure 2B). The experimental cells were divided into five groups: control group, miR-148b-3p (+) NC group, miR-148b-3p (+) group, miR-148b-3p (−) NC group, and miR-148b-3p (−) group.

The stable transfected HOTAIR knockdown cells were transiently co-transfected with miR-148b-3p agomir, miR-148b-3p antagomir, or their relevant NC. The experiment cells were divided into five groups: control group, HOTAIR (−) NC + miR-148b-3p (+) NC group, HOTAIR (−) + miR-148b-3p (+) group, HOTAIR (−) NC + miR-148b-3p (−) NC group, and HOTAIR (−) + miR-148b-3p (−) group.

The stable transfected USF1 overexpression cells were transiently co-transfected with miR-148b-3p agomir or relevant NC. The experiment cells were divided into five groups: control group, miR-148b-3p (+) NC + USF1 (+) NC group, miR-148b-3p (+) + USF1 (+) NC group, miR-148b-3p (+) NC + USF1 (+) group and miR-148b-3p (+) + USF1 (+) group.

### Transendothelial electric resistance (TEER) and horseradish peroxidase (HRP) flux assays

TEER measurement was performed to measure the integrity of the BTB. Firstly, the BTB model *in vitro* was established successfully. Then, TEER-values were measured with millicell-ERS apparatus (Millipore, Billerica, MA, USA). To ensure temperature equilibration and the same medium composition, Transwell inserts were placed at room temperature for 30 min and the mediums were refreshed before measurement. Background electrical resistance was subtracted from each reading when the final resistance was calculated. The final results were expressed as Ω•cm^2^, according to the surface area of Transwell inserts.

HRP flux (HRP, 0.5 μM, Sigma-Aldrich, USA) was detected to further measure the permeability of the BTB *in vitro*. After BTB models were constructed, HRP was added to the upper chamber of Transwell inserts. The working concentration of HRP was 10 μg/ml. One hour later, 5 μl of culture medium was collected from the lower chamber of Transwell inserts. The HRP content was measured with a spectrophotometer using TMB colorimetry. The final HRP flux was expressed as pmol/cm^2^/h.

### Quantitative real-time PCR assay (qRT-PCR)

The expression levels of HOTAIR and miR-148b-3p were detected by qRT-PCR. All qRT-PCR analyses were conducted by means of a 7500 Fast Real-Time PCR System (Applied Biosystems, Foster City, CA, USA). Total RNA was extracted from ECs, GECs and transfected cells using Trizol reagent (Life Technologies Corporation, Carlsbad, CA, USA) by the manufacturer's instructions. The RNA concentration and quality were determined by the NanoDrop Spectrophotometer (ND-100; NanoDrop, Wilmington, DE). Primers of HOTAIR were as follows: forward: 5′-GGT AGA AAA AGC AAC CAC GAA GC-3′; reverse: 5′-ACA TAA ACC TCT GTC TGT GAG TGC C-3′. Quantitative RT-PCR of HOTAIR was conducted using One Step SYBR® Primer Script™ RT-PCR Kit (TaKaRa, Dalian, China) according to the manufacturer's instructions. The expression level of HOTAIR was normalized to that of GAPDH (forward: 5′-GGTGAAGGTCGGAGTCAACG-3′; reverse: 5′-CCATGTAGTTGAGGTCAATGAAG-3′) with the relative quantification 2^−ΔΔCt^ formula. TaqMan® MicroRNA Reverse Transcription Kit (Applied Biosystems, Foster City, CA, USA) was used for miR-148b-3p reverse transcription. Real-time PCR analysis was performed using TaqMan® Universal Master Mix II (Applied Biosystems, Foster City, CA, USA). The probes of miR-148b-3p (000471) and U6 (001973) were used. The expression level of miR-148b-3p was normalized to that of U6 with the relative quantification 2^−ΔΔCt^ formula.

### Western blot assay

The protein expression levels of USF1 and tight junction related proteins were detected by western blot analysis. Cells total proteins were extracted in RIPA buffer (Beyotime Institute of Biotechnology, Jiangsu, China) with protease inhibitors PMSF. The protein concentrations were determined by the BCA protein assay kit (Beyotime Institute of Biotechnology, Jiangsu, China). Equal amounts of proteins were separated with SDS-PAGE and transferred onto polyvinylidene fluoride (PVDF) membranes (Millipore, USA). Non-specific bindings of the membranes were blocked with 5% fat-free milk in TTBS for 2 h and then incubated with primary antibodies for USF1 (diluted 1:500; Santa Cruz Biotechnology, Santa Cruz, CA, USA), ZO-1 (diluted 1:300; Life Technologies Corporation, Frederick, MD, USA), occludin (diluted 1:600; Abcam, Cambridge, MA, USA), claudin-5 (diluted 1:300; Life Technologies Corporation, Frederick, MD, USA), and GAPDH (diluted 1:10,000; Proteintech, USA) at 4°C overnight. The membranes were washed three times with TTBS and subsequently incubated with respective HRP-conjugated secondary antibody at room temperature for 2 h. Protein bands were visualized by enhanced chemiluminescence (ECL, Santa Cruz Biotechnology, USA) and scanned using the Chemi Imager 5500 V2.03 software (AlPha Innotech, San Leandro, CA, USA). Relative integrated light density values (IDVs) of bands were calculated by the Fluor chen 2.0 software (Alpha Innotech, San Leandro, CA, USA) and normalized with those of GAPDH.

### Immunofluorescence assay

In order to detect the expression and distribution of tight junction related proteins, immunofluorescence assay was performed. The cells cultured on insert filters should be at 100% confluence and fixed with 4% paraformaldehyde at room temperature for 20 min (ZO-1 and claudin-5) or fixed with methanol for 10 min at −20°C (occludin). Then the cells were permeabilized with 0.2% Triton X-100 for 10 min and blocked with 5% BSA for 2 h at room temperature. The cells were incubated with primary antibodies against ZO-1, occludin, and claudin-5 at 4°C overnight. All the antibodies were diluted at 1:50. The cells were washed with PBST for three times and incubated with Alexa Fluor 555-labeled anti-rabbit IgG or anti-mouse IgG secondary antibodies (diluted 1:500; Beyotime Institute of Biotechnology, Jiangsu, China) for 2 h in dark room. The nuclei were stained with 0.5 μg/ml DAPI for 5–8 min. The staining were visualized by immunofluorescence microscopy (Olympus, Tokyo, Japan) and the images were merged with Chemi Imager 5500 V2.03 software.

### Dual-luciferase reporter assays

The miR-148b-3p binding sites of HOTAIR were predicted with the help of computer-aided algorithms: starbase 2.0 (http://starbase.sysu.edu.cn). The miR-148b-3p binding sites of USF1 were predicted by TargetScan (http://www.targetscan.org). To examine whether miR-148b-3p targeted HOTAIR and USF1 directly, wild-type HOTAIR reporter plasmid (HOTAIR wt), mutated-type HOTAIR reporter plasmid (HOTAIR mut), wild-type USF1 3′UTR reporter plasmid (USF1 wt), and mutated-type USF1 3′UTR reporter plasmid (USF1 mut) were constructed with pmirGLO-promoter vector by Generay Biotechnology (Shanghai, China). For instance, the fragment of HOTAIR containing the putative miR-148b-3p binding sites was subcloned into pmirGLO Dual-Luciferase miRNA Target Expression Vector to form the reporter vector HOTAIR-wild-type (HOTAIR wt). To test the binding specificity, the corresponding mutants of putative miR-148-3p binding sites were created to form the reporter vector HOTAIR-mutated-type (HOTAIR mut). HEK 293T cells seeded in 96-well plates at 60–80% confluence were co-transfected with wild-type or mutated-type pmirGLO-HOTAIR (pmirGLO-USF1) reporter plasmid and miR-148b-3p agomir or agomir-NC using lipofectamine 3000. After 48 h, the luciferase activity was analyzed using the Dual-Luciferase Reporter Assay System (Promega, Madison, WI, USA). The relative luciferase activity was expressed as the ratio of firefly luciferase activity to renilla luciferase activity.

### Chromatin immunoprecipitation (ChIP) assay

To clarify whether USF1 bound to the promoters of tight junction related proteins, ChIP assay was performed. Simple ChIP Enzymatic Chromatin IP Kit (Cell signaling Technology, Danvers, Massachusetts, USA) was used according to the manufacturer's instruction. In brief, cells were crosslinked with 1% formaldehyde for 10 min and treated with glycine for 5 min. Cells were collected in cold lysis buffer containing PMSF. Chromatin was digested by Micrococcal Nuclease for 20 min at 37°C. Before adding antibody 2% input reference was removed and stored at −20°C. Three micrograms of anti-USF1 antibody (Santa Cruz Biotechnology, CA, USA) was added in the immunoprecipitation sample with gentle shaking at 4°C overnight. Negative control was conducted with normal rabbit IgG. The chromatinimmune complex was eluted from the antibody/Protein G beads with gentle vortexing at 65°C for 30 min.

The DNA crosslinks was reversed by 5 mol/L NaCl and Proteinase K at 65°C for 2 h and DNA was purified. PCR was performed to amplify immunoprecipitated DNA. The detail informations of specific primers were listed in Table 1.

**Table 1:** Primers used for ChIP assay.

**Gnen**	**Control and binding side**	**Sequences**	**Product size (bp)**	**Annealing temperature (°C)**
ZO-1	PCR1	(F)G TCAGTGCATTTGTAGATAGTGTC	135	50
		(R)AAAGGTGGTGATGAAAGACCT		
	PCR2	(F)GTCTAGGATTGGTTTCTTACCATGT	207	48
		(R)GGCCATCAAGATTGCTGAA		
Occludin	PCR1	(F)CACATTCCCACCAACAGACTT	237	51
		(R)CCTGCAGTCAAATGGATAAGATG		
	PCR2	(F)AAAACCCACTGAATTGTACGTG	237	50
		(R)AATCCCCTTAATGTTCCCTGT		
Claudin-5	PCR1	(F)CACCTCTGGGATCTTGCACT	119	53
		(R)AGAACTGGGCAGGAAAGACA		
	PCR2	(F)CCAGGAGGGTCTGTAGAGGA	165	49
		(R)TGAGGCTGGAAGGAAATCA		

### Statistical analysis

Statistical analysis was performed using SPSS 19.0 statistical software. Data was described as mean ± SD. Student's *t*-test was used to analyze the difference between two groups. One-way analysis of variance (ANOVA) followed by Dunnett's post-test was used to analyze the difference among multiple groups. *P* < 0.05 was considered to be statistically significant.

## Results

### The endogenous expressions of HOTAIR, miR-148b-3p, and USF1 in ECs and GECs

As shown in Figure 1, “ECs” means normal endothelial cells, yet “GECs” means glioma microvascular endothelial cells. The relative expressions of HOTAIR and miR-148b-3p were detected by qRT-PCR analysis. Compared with ECs group, the expression of HOTAIR was significantly up-regulated (*P* < 0.01; Figure 1A), but miR-148b-3p was down-regulated in GECs group (*P* < 0.05; Figure 1B). Besides, western blot assay demonstrated the expression of USF1 was significantly up-regulated in GECs group compared with ECs group (*P* < 0.01; Figure 1C).

### Knockdown of HOTAIR significantly increased BTB permeability and decreased the expressions of tight junction related proteins as well as changed the distribution of these proteins in GECs

As shown in Figure 2, un-transfected GECs group marked as “Control” group, stable transfected GECs with shHOTAIR marked as “HOTAIR (−)” group and its NC marked as “HOTAIR (−) NC” group. The stable transfected cells was acquired after G418 screening. TEER and HRP flux were performed to evaluate the permeability of BTB after the BTB models were established. As shown in Figure 2A, TEER-value of HOTAIR (−) group was significantly lower than HOTAIR (−) NC group (*P* < 0.05). But there was no statistical difference between control and HOTAIR (−) NC groups (*P* > 0.05). The results of HRP flux were shown in Figure 2B, the penetration rate of HRP in HOTAIR (−) group was higher than that of HOTAIR (−) NC group (*P* < 0.01); however, there was no significant difference between control and HOTAIR (−) NC groups (*P* > 0.05).

**Figure 2:** HOTAIR regulated the permeability of BTB *in vitro* and the expressions of tight junction related proteins in GECs. **(A)** TEER-values of GECs were expressed as Ω•cm^2^. Data represent means ± SD (*n* = 4, each group). ^*^P < 0.05 vs. HOTAIR (–) NC group. **(B)** HRP flux was calculated as pmol/cm^2^/h. Data represent means ± SD (*n* = 5, each group). ^**^P < 0.01 vs. HOTAIR (–) NC group. **(C,D)** Western blot analysis of tight junction related proteins ZO-1, occludin, and claudin-5 in GECs. The IDVs of protein expressions were shown using GAPDH as an endogenous control. Data represent mean ± SD (*n* = 3, each group). ^**^P < 0.01 vs. HOTAIR (–) NC group. **(E)** Immunofluorescence localization of ZO-1, occludin, and claudin-5 in GECs. ZO-1 (red), occludin (red), and claudin-5 (red) were, respectively, labeled with fluorescent secondary antibody and nuclei were labeled with DAPI. Images were representative of three independent experiments. Scale bar = 20 μm.

In addition, the expressions of tight junction related proteins ZO-1, occludin, and claudin-5 in GECs were significantly down-regulated in the HOTAIR (−) group compared with the HOTAIR (−) NC group (*P* < 0.01); while their expressions showed no significant difference between control and HOTAIR (−) NC groups (*P* > 0.05; Figures 2C,D). Immunofluorescence analysis was shown in Figure 2E, In control and HOTAIR (−) NC groups, ZO-1, occludin, and claudin-5 displayed a continuous distribution at the edge of GECs; yet the immune response of ZO-1, occludin, and claudin-5 in HOTAIR (−) group were weakened than in HOTAIR (−) NC group and these proteins exhibited a discontinuous distribution at the edge of GECs.

### Knockdown of HOTAIR increased the expression of miR-148b-3p and decreased the expression of USF1

The expressions of miR-148b-3p and USF1 were detected after BTB models were established with stable transfected cells. As shown in Figure 3A, the expression of miR-148b-3p in HOTAIR (−) group was significantly increased compared with HOTAIR (−) NC group (*P* < 0.05); however, there was no statistical difference between control and HOTAIR (−) NC group (*P* > 0.05). As shown in Figure 3B, the expression of USF1 was significantly decreased in HOTAIR (−) group (*P* < 0.05), compared with HOTAIR (−) NC group; while there was no significant difference between control and HOTAIR (−) NC groups (*P* > 0.05).

**Figure 3:** HOTAIR regulated the expressions of miR-148b-3p and USF1 in GECs. **(A)** The relative expression level of miR-148b-3p in GECs was detected by qRT-PCR. Data represent mean ± SD (*n* = 3, each group). ^*^P < 0.05 vs. HOTAIR (–) NC group. **(B)** The protein expression of USF1 was shown by western blot. The IDVs of USF1 were shown using GAPDH as an endogenous control. Data represent mean ± SD (*n* = 3, each group). ^*^P < 0.05 vs. HOTAIR (–) NC group.

### Knockdown of HOTAIR decreased the expressions of USF1 and tight junction related proteins and increased the permeability of BTB through the negative regulation of miR-148b-3p

As shown in Figure 4, there are five groups: “Control” means un-transfected GECs, “HOTAIR (−) NC + miR-148b-3p (+) NC” means stable transfected GECs of shHOTAIR NC was transiently transfected with miR-148b-3p agomir NC; “HOTAIR (−) + miR-148b-3p (+)” means stable transfected GECs of shHOTAIR was transiently transfected miR-148b-3p agomir; “HOTAIR (−) NC + miR-148b-3p (−) NC” means stable transfected GECs of shHOTAIR NC was transiently transfected with miR-148b-3p antagomir NC; “HOTAIR (−) + miR-148b-3p (−)” means stable transfected GECs of shHOTAIR was transiently transfected miR-148b-3p antagomir.

**Figure 4:** Knockdown of HOTAIR increased BTB permeability as well as decreased the expressions of tight junction related proteins and USF1 in GECs by negatively regulating miR-148b-3p. **(A)** TEER-values of GECs were expressed as Ω•cm^2^. Data represent mean ± SD (*n* = 4, each group). **(B)** HRP flux was calculated as pmol/cm^2^/h. Data represent mean ± SD (*n* = 4, each group). **(C–F)** Western blot analysis of tight junction related proteins and USF1 in GECs. The IDVs of protein expressions were shown using GAPDH as an endogenous control. Data represent mean ± SD (*n* = 3, each group). ^*^P < 0.05 and ^**^P < 0.01 vs. HOTAIR (−) NC + miR-148b-3p (+) NC group.

As shown in Figure 4A, TEER-value of HOTAIR (−) + miR-148b-3p (+) group was significantly lower than that of HOTAIR (−) NC + miR-148b-3p (+) NC group (*P* < 0.05); but compared with HOTAIR (−) NC + miR-148b-3p (−) NC group, TEER-value of HOTAIR (−) + miR-148b-3p (−) group had no statistical difference (*P* > 0.05); and TEER-values of HOTAIR (−) NC+miR-148b-3p (+) NC and HOTAIR (−) NC + miR-148b-3p (−) NC groups were not statistically significant compared with control group (*P* > 0.05). As shown in Figure 4B, the changes of HRP flux were contrary to TEER-values. Compared with HOTAIR (−) NC + miR-148b-3p (+) NC group, HRP flux in HOTAIR (−) + miR-148b-3p (+) group was increased significantly (*P* < 0.01); while compared with HOTAIR (−) NC + miR-148b-3p (−) NC group, HRP flux in HOTAIR (−) + miR-148b-3p (−) group had no statistical difference (*P* > 0.05); and there was no significant difference among control, HOTAIR (−) NC + miR-148b-3p (+) NC and HOTAIR (−) NC + miR-148b-3p (−) NC groups (*P* > 0.05).

Moreover, the expressions of tight junction related proteins ZO-1, occludin, and claudin-5 (Figures 4C,D) as well as USF1 (Figures 4E,F) were significantly down-regulated in HOTAIR (−) + miR-148b-3p (+) group (*P* < 0.01) compared with HOTAIR (−) NC + miR-148b-3p (+) NC group; but the expressions of these proteins in HOTAIR (−) + miR-148b-3p (−) group were not statistically significant compared with HOTAIR (−) NC + miR-148b-3p (−) NC groups (*P* > 0.05); and there was no significant difference among control, HOTAIR (−) NC + miR-148b-3p (+) NC and HOTAIR (−) NC + miR-148b-3p (−) NC groups (*P* > 0.05).

### HOTAIR was a target RNA of miR-148b-3p

There are five groups in Figure 5: “Control” means pmirGLO blank vector, “miR-148b-3p (+) NC + HOTAIR wt” means co-transfection of miR-148b-3p agomir NC and wild-type HOTAIR reporter plasmid; “miR-148b-3p (+) + HOTAIR wt” means co-transfection of miR-148b-3p agomir and wild-type HOTAIR reporter plasmid; “miR-148b-3p (+) NC + HOTAIR mut” means co-transfection of miR-148b-3p agomir NC and mutated-type HOTAIR reporter plasmid; “miR-148b-3p (+) + HOTAIR mut” means co-transfection of miR-148b-3p agomir and mutated-type HOTAIR reporter plasmid.

**Figure 5:** The interaction between lncRNA HOTAIR and miR-148b-3p was detected by dual-luciferase reporter assay. Relative luciferase activity was expressed as firefly/renilla luciferase activity. Data represent mean ± SD (*n* = 3, each group). ^**^P < 0.01 vs. miR-148b-3p (+) NC + HOTAIR wt group.

The miR-148b-3p binding sites of HOTAIR were predicted with the help of computer-aided algorithms: starbase 2.0 (http://starbase.sysu.edu.cn). The results of dual-luciferase reporter assay were shown in Figure 5. Compared with miR-148b-3p (+) NC + HOTAIR wt group, the relative luciferase activity in miR-148b-3p (+) + HOTAIR wt group was significantly decreased (*P* < 0.01). However, compared with miR-148b-3p (+) NC + HOTAIR mut group, the relative luciferase activity showed no significant difference in comparison with miR-148b-3p (+) + HOTAIR mut groups (*P* > 0.05).

### miR-148b-3p regulated BTB permeability and affected the expressions of USF1 and tight junction related proteins in GECs

As shown in Figure 6, there are five groups: “Control” means un-transfected GECs, “miR-148b-3p (+) NC” means transiently transfected GECs with miR-148b-3p agomir NC; “miR-148b-3p (+)” means transiently transfected GECs with miR-148b-3p agomir; “miR-148b-3p (−) NC” means transiently transfected GECs with miR-148b-3p antagomir NC; “miR-148b-3p (−)” means transiently transfected GECs with miR-148b-3p antagomir.

**Figure 6:** miR-148b-3p regulated BTB permeability as well as the expressions of USF1 and tight junction related proteins in GECs. **(A)** miR-148b-3p changed TEER-values of GECs. **(B)** miR-148b-3p changed HRP flux of GECs **(C–F)** miR-148b-3p modulated the protein expressions of USF1 and tight junction related proteins in GECs. The IDVs of protein expressions were shown using GAPDH as an endogenous control. **(G)** Immunofluorescence localization of ZO-1, occludin, and claudin-5 in GECs. ZO-1 (red), occludin (red), and claudin-5 (red) were, respectively, labeled with fluorescent secondary antibody and nuclei were labeled with DAPI. Images were representative of five independent experiments. Scale bar = 20 μm. Data represent mean ± SD (*n* = 3, each group). ^*^P < 0.05 vs. miR-148b-3p (+) NC group. ^*##*^*P* < 0.01 and ^#^*P* < 0.05 vs. miR-148b-3p (–) NC group.

As shown in Figure 6A, TEER-value in the miR-148b-3p (+) group was significantly decreased compared with miR-148b-3p (+) NC group (*P* < 0.05); conversely, TEER-value in the miR-148b-3p (−) group was significantly increased compared with miR-148b-3p (−) NC group (*P* < 0.01). And compared with control group, TEER-value had no significant difference in miR-148b-3p (+) NC and miR-148b-3p (−) NC groups (*P* > 0.05). The results of HRP flux were shown in Figure 6B, the penetration rate of HRP in the miR-148b-3p (+) group was significantly increased compared with miR-148b-3p (+) NC group (*P* < 0.05); however, the penetration rate of HRP in the miR-148b-3p (−) group was significantly decreased compared with miR-148b-3p (−) NC group (*P* < 0.05). Meanwhile, compared with control group, the penetration rate of HRP had no significant difference in miR-148b-3p (+) NC and miR-148b-3p (−) NC groups (*P* > 0.05).

The protein expressions of USF1 (Figures 6C,D) and tight junction related proteins ZO-1, occludin, and claudin-5 (Figures 6E,F) in GECs were shown in Figure 6. Compared with miR-148b-3p (+) NC group, the expressions of these proteins in the miR-148b-3p (+) group were significantly decreased (*P* < 0.05). On the contrary, compared with miR-148b-3p (−) NC group, the expressions of these proteins were significantly increased in the miR-148b-3p (−) group (*P* < 0.05). But there was no significant difference among control, miR-148b-3p (+) NC and miR-148b-3p (−) NC groups (*P* > 0.05).

Immunofluorescence analysis was shown in Figure 6G. Tight junction related proteins ZO-1, occludin, and claudin-5 displayed a continuous distribution at the edge of GECs in control, miR-148b-3p (+) NC, and miR-148b-3p (−) NC groups. Compared with miR-148b-3p (+) NC group, immune response of ZO-1, occludin, and claudin-5 were weakened and exhibited a discontinuous distribution in the miR-148b-3p (+) group. Compared with miR-148b-3p (−) NC group, immune response of ZO-1, occludin, and claudin-5 were enhanced and exhibited a continuous distribution in the miR-148b-3p (−) group.

### miR-148b-3p regulated BTB permeability as well as the expression of USF1 and tight junction related proteins by negative regulation of USF1

Stable transfected USF1 overexpression GECs (screening with G418 after transfected with lipo2000) were used to establish BTB models first and were transiently transfected with miR-148b-3p agomir or its NC. As shown in Figure 7, there are five groups: “Control” means un-transfected GECs, “miR-148b-3p (+) NC + USF1 (+) NC” means stable transfected USF1 overexpression NC GECs were transiently transfected with miR-148b-3p agomir NC; “miR-148b-3p (+) + USF1 (+) NC” means stable transfected USF1 overexpression GECs were transiently transfected with miR-148b-3p agomir; “miR-148b-3p (+) NC + USF1 (+)” means stable transfected USF1 overexpression NC GECs were transiently transfected with miR-148b-3p agomir; “miR-148b-3p (+) + USF1 (+)” means stable transfected USF1 overexpression GECs were transiently transfected with miR-148b-3p agomir. The changes of TEER-values and HRP flux were detected after 48 h. As shown in Figure 7A, compared with miR-148b-3p (+) NC + USF1 (+) NC group, TEER-value of miR-148b-3p (+) + USF1 (+) NC group was significantly decreased (*P* < 0.01), but that of miR-148b-3p (+) NC + USF1 (+) group was increased remarkably (*P* < 0.01). Compared with miR-148b-3p (+) + USF1 (+) NC group, TEER-value of miR-148b-3p (+) + USF1 (+) group was dramatically increased (*P* < 0.01). And there was no significant difference between control and miR-148b-3p (+) NC + USF1 (+) NC (*P* > 0.05). As shown in Figure 7B, compared with miR-148b-3p (+) NC + USF1 (+) NC group, the penetration rate of HRP in miR-148b-3p (+) + USF1 (+) NC group was significantly increased (*P* < 0.01), however, that in miR-148b-3p (+) NC + USF1 (+) group was significantly decreased (*P* < 0.05). Compared with miR-148b-3p (+) + USF1 (+) NC group, the penetration rate of HRP in miR-148b-3p (+) + USF1 (+) group significantly decreased (*P* < 0.05). And there was no significant difference between control and miR-148b-3p (+) NC + USF1 (+) NC group (*P* > 0.05).

**Figure 7:** miR-148b-3p regulated BTB permeability as well as the expressions of USF1 and tight junction related proteins in GECs by inhibiting of USF1. **(A)** TEER-values of GECs were detected expressed as Ω•cm^2^. **(B)** HRP flux was performed and calculated as pmol/cm^2^/h. **(C,D)** The protein expressions of USF1 and tight junction related proteins in GECs were detected by western blot. The IDVs of protein expression levels were shown using GAPDH as an endogenous control. Data represent mean ± SD (*n* = 3, each group). ^*^P < 0.05 and ^**^P < 0.01 vs. miR-148b-3p (+) NC + USF1 (+) NC group, ^#^*P* < 0.05 and ^*##*^*P* < 0.01 vs. miR-148b-3p (+) + USF1 (+) NC group.

Simultaneously, the expressions of USF1 and tight junction related proteins ZO-1, occludin, and claudin-5 were shown in Figures 7C,D. Compared with miR-148b-3p (+) NC + USF1 (+) NC group, the expressions of these proteins in miR-148b-3p (+) + USF1 (+) NC group were significantly down-regulated (*P* < 0.01), but that in miR-148b-3p (+) NC + USF1 (+) group were significantly up-regulated (*P* < 0.01). Compared with miR-148b-3p (+) + USF1 (+) NC group, the expressions of these proteins in miR-148b-3p (+) + USF1 (+) group significantly up-regulated (*P* < 0.01). Yet there was no significant difference between control and miR-148b-3p (+) NC + USF1 (+) NC group (*P* > 0.05).

### USF1 was a target of miR-148b-3p

There are five groups in Figure 8: “Control” means pmirGLO blank vector, “miR-148b-3p (+) NC + USF1 wt” means co-transfection of miR-148b-3p agomir NC and wild-type USF1 reporter plasmid; “miR-148b-3p (+) + USF1 wt” means co-transfection of miR-148b-3p agomir and wild-type USF1 reporter plasmid; “miR-148b-3p (+) NC + USF1 mut” means co-transfection of miR-148b-3p agomir NC and mutated-type USF1 reporter plasmid; “miR-148b-3p (+) + USF1 mut” means co-transfection of miR-148b-3p agomir and mutated-type USF1 reporter plasmid.

**Figure 8:** USF1 was a target of miR-148b-3p. Relative luciferase activity was performed by dual-luciferase reporter assay. Relative luciferase activity was expressed as firefly/renilla luciferase activity. Data represent mean ± SD (*n* = 3, each group). ^*^P < 0.05 vs. miR-148b-3p NC + USF1 wt group.

The miR-148b-3p binding sites of USF1 were predicted by bioinformatics software TargetScan 7.1 (http://www.targetscan.org). The results of dual-luciferase reporter assay were shown in Figure 8. Compared with miR-148b-3p (+) NC + USF1 wt group, the relative luciferase activity in miR-148b-3p (+) + USF1 wt group was significantly decreased (*P* < 0.05). Whereas, the relative luciferase activity in miR-148b-3p (+) + USF1 mut demonstrated no significant difference compared with miR-148b-3p (+) NC + USF1 mut group (*P* > 0.05).

### USF1 regulated BTB permeability and the expressions of tight junction related proteins ZO-1, occludin, and claudin-5 in GECs

There are five groups in Figure 9: “Control” means un-transfected GECs, “USF1 (+) NC” means stable transfected GECs with USF1 overexpression plasmid NC; “USF1 (+)” means stable transfected GECs with USF1 overexpression plasmid; “USF1 (−) NC” means stable transfected GECs with USF1 silence plasmid NC; “USF1 (−)” means stable transfected GECs with USF1 silence plasmid. The transfection efficiencies of USF1 overexpression and silence were validated as 74.8 and 62.6%, respectively, as shown in Figures 9A,B. Compared with USF1 (+) NC group, TEER-value of USF1 (+) group was significantly higher (*P* < 0.05; Figure 9C). And compared with USF1 (−) NC group, TEER-value of USF1 (−) group was significantly lower (*P* < 0.01). Whereas, there was no statistical difference among control, USF1 (+) NC and USF1 (−) NC groups (*P* > 0.05). Numerically, the trends of HRP flux were opposite to the result of TEER as shown in Figure 9D. Compared with USF1 (+) NC group, the penetration rate of HRP in USF1 (+) group was significantly reduced (*P* < 0.01). Compared with USF1 (−) NC group, that of HRP in USF1 (−) group was significantly increased (*P* < 0.01). And there was no statistical difference among control, USF1 (+) NC, and USF1 (−) NC groups (*P* > 0.05).

**Figure 9:** USF1 regulated BTB permeability and the expressions of tight junction related proteins in GECs. **(A,B)** The protein expression of USF1 was assessed by western blot to validate the efficiency of transfection. GAPDH was used as an endogenous control. **(C)** TEER-values of GECs were detected after USF1 overexpression and silencing. **(D)** HRP flux was performed after USF1 overexpression and silencing. **(E,F)** The protein expressions of tight junction related proteins in GECs were detected after USF1 overexpression and silencing. The IDVs of protein expression levels were shown using GAPDH as an endogenous control. Data represent mean ± SD (*n* = 3, each group). ^*^P < 0.05 and ^**^P < 0.01 vs. USF1 (+) NC group, ^*##*^*P* < 0.01 vs. USF1 (–) NC group.

Additionally, the expressions of tight junction related proteins ZO-1, occludin, and claudin-5 in GECs of USF1 (+) group were significantly increased compared with USF1 (+) NC group (*P* < 0.05; Figures 9E,F). And their expressions of USF1 (−) group were significantly reduced compared with USF1 (−) NC group (*P* < 0.01). Whereas, there was no statistical difference among control, USF1 (+) NC and USF1 (−) NC groups (*P* > 0.05).

### USF1 bound to the promoters of tight junction related proteins *ZO-1, occludin*, and *claudin-5*

Eventually, ChIP assays were performed to clarify whether USF1 are directly associated with the promoters of *ZO-1, occludin*, and *claudin-5*. The Potential binding sites were predicted by bioinformatics software DBTSS HOME (http://dbtss.hgc.jp/) and the “TFSEARCH” program (http://mbs.cbrc.jp/reach/db/TFREARCH). We analyzed the potential binding sites of DNA sequences of upstream region 3,000 bp and downstream region 200 bp from the position of transcription start site (TSS) of *ZO-1, occludin*, and *claudin-5*. A putative USF1 binding sites at −786 bp position in *ZO-1*, a putative USF1 binding sites at −1,154 bp position in *occludin* and one putative USF1 binding sites at −644 bp position in *claudin-5* were, respectively, confirmed. Specific primers were designed according to the putative USF1 binding sequence and NC s were designed too. The results revealed that there were associations of USF1 with putative binding sites (CACGTG) of *ZO-1* (Figure 10A, CATGTG) of *occludin* (Figure 10B) and (CACGTG) of *claudin-5* (Figure 10C), but no relationships with all of the NC groups.

**Figure 10:** USF1 bound to the promoters of tight junction related proteins in GECs. **(A–C)** Schematic representation of the human *ZO-1*, *occludin*, and *claudin-5* promoter regions in 3,000 bp upstream of the transcription start site (TSS, designated as +1). CHIP PCR products for binding sites and upstream regions not expected to associate with USF1 were amplified by PCR using their specific primers. Images were representative of three independent CHIP experiments.

## Discussion

Recent studies showed lncRNAs were not only closely related to the development and progression of cancers, but also involved in the regulation of vascular endothelial cell function (Xu et al., 2014). TUG1 and MALAT1, as lncRNAs, were up-regulated in GECs and were involved in regulating the permeability of BTB (Cai et al., 2015a; Ma et al., 2016). HOTAIR, ~2,158 nucleotides in length, existed in the genome sequence of mammals and located between HOXC11 and HOXCl2 in chromosome 12q13.13 (He et al., 2011). It has been reported that HOTAIR could influence methylation of histone, resulting in silence of target genes (Grier et al., 2005; Tsai et al., 2010). HOTAIR was highly expressed in many cancer tissues and exerted the role of oncogene (Gupta et al., 2010; Geng et al., 2011; Hajjari et al., 2013; Kim et al., 2013; Zhang et al., 2013; Zhuang et al., 2013). HOTAIR was highly expressed in malignant gliomas tissues or U87 and U251 cells, and silence of HOTAIR decreased the abilities of proliferation, migration, and invasion as well as promoted cell apoptosis in glioma cells, and these influences on the biological behavior of glioma cells were achieved through the competitive inhibition of HOTAIR on miR-326-mediated targeting combination with FGF1 (Ke et al., 2015). In kidney cancer, miR-141 targeted to HOTAIR and suppressed HOTAIR expression to inhibit the proliferation and invasion of tumor cells (Chiyomaru et al., 2014). This study found HOTAIR expression was up-regulated in GECs for the first time. Overexpression of HOTAIR in tumor vascular endothelial cells was also existed in nasopharynx cancer, cervical cancer, and breast cancer (Li et al., 2014; Kim et al., 2015; Fu et al., 2016). Our findings further revealed HOTAIR knockdown in GECs significantly increased the permeability of BTB, which implying HOTAIR might regulate the function of GECs and thereby change the permeability of BTB.

Usually, miRNAs could specially bind to 3′-UTR of target messenger RNA (mRNA) and negatively regulate the expression of target gene (Lewis et al., 2005). MiR-148b-3p was located in chromosome 12q13.13, and its expression was down-regulated in many cancer tissues. For example, miR-148b expression was decreased in hepatocellular carcinoma tissues, which could considerably be linked to malignant clinical pathological index, such as vascular invasion and TNM stage (Zhang Z. et al., 2014). MiR-148b inhibited the proliferation and invasion of pancreatic cancer cells by targeting AMPKa1, and acted as a tumor suppressor in the development and progression of pancreatic cancer (Bloomston et al., 2007). The expression of miR-148b was significantly down-regulated in colorectal cancer tissues compared with non-tumor adjacent tissues. The overexpression of miR-148b inhibited the proliferation of colorectal cancer (Song et al., 2012). Besides, the expression of miR-148b in gastric cancer tissue was significantly lower than its surrounding non-tumor tissues and the lower expression of miR-148b was related to the size and Borrmann types of the tumor (Song et al., 2011). The present study highlighted the expression of miR-148b-3p in GECs was declined compared with normal ECs. The overexpression of miR-148b-3p reduced the expression of tight junction related proteins ZO-1, occludin, and claudin-5 and increased of BTB permeability. Above results suggested miR-148b-3p played important roles in the regulation of BTB permeability. Our previous studies unveiled the effects and mechanisms of certain miRNA on BTB permeability, for example, miR-181a targeting KLF6, miR-18a targeting RUNX1, and miR-34c targeting MAZ significantly regulated BTB permeability, respectively (Ma et al., 2014b; Miao et al., 2015; Zhao L. et al., 2015).

In order to further investigate target combination between HOTAIR and miR-148b-3p, bioinformatics software predicted the potential binding sites of miR-148b-3p in HOTAIR mRNA, which were verified by dual luciferase reporter assay. Our findings also revealed knockdown of HOTAIR reduced the expressions of ZO-1, occludin, and claudin-5 in GECs and finally increased the permeability of BTB by targeting miR-148b-3p. Wang's research about miR-148b-3p inhibits malignant biological behaviors of human glioma cells induced by high HOTAIR expression supports our results (Wang G. et al., 2016). These research indicated HOTAIR might play an important regulatory role either in glioma cells or GECs by targeting miR-148b-3p.

Recent studies reported miR-148b-3p influenced the response of lung adenocarcinoma cell to hypoxia by targeting NOG and WNT10B (Geng et al., 2016). miR-148b inhibited the proliferation of gastric cancer cells by targeting CCKBR (Song et al., 2011) and inhibited the growth of rectal cancer cells by targeting CCK2R (Song et al., 2012). Besides, miR-148b promoted aberrant glycosylation of IgA1 in IgA nephropathy via targeting C1GALT1 (Serino et al., 2012). USF, as an important transcription factor, consisted of two main genes, USF1 and USF2, which ubiquitously existed in eukaryotes and had highly conserved bHLH-LZ domain and bound to consensus sequence CANNTG of E-box to regulate the gene transcription (Allen et al., 2005; Rada-Iglesias et al., 2008). USF took part in various gene regulations, such as stress, immune response, cell cycle and proliferation, fat and carbohydrate metabolism, and ultraviolet ray activation associated with chromatosis (Corre and Galibert, 2005). The present study demonstrated the expression of USF1 in GECs was increased significantly and USF1 was a target of miR-148b-3p. Simultaneously, overexpression of both USF1 and miR-148b-3p showed the overexpression of USF1 could effectively reverse miR-148b-3p mediated up-regulation on BTB permeability, which pointing out that miR-148b-3p increased BTB permeability by negatively regulating USF1. There were similar studies about miRNA regulating transcription factor to change BTB permeability: miR-18a targeting RUNX1 (Miao et al., 2015) as well as miR-34a targeting PKCε could regulate BTB permeability significantly (Zhao W. et al., 2015).

There were two pathways to regulate the permeability of BTB: para-cellular pathway and transcellular pathway (Fan et al., 2011). Tight junction related protein family were the crucial proteins for transcellular pathway, including membrane cytoskeletal proteins zonula occludens (ZO-1 and ZO-2), transmembrane proteins occludin and claudins, adhesion molecules (JAM), and so on (Abbott, 2013). ZO-1, a member of guanylate kinase-like proteins family, is located on the surface of cytoplasmic membrane. Occludin and claudin-5, as integral membrane proteins of endothelial cells, constitute tight junctions between the adjacent cells and were connected with cytoskeletal protein by ZO-1 to accordingly maintain the integrity and permeability of BBB (Aijaz et al., 2006; Luissint et al., 2012). A great amount of studies reported the down-regulated expressions of tight junction related proteins ZO-1, occludin, and claudin-5 increased BTB permeability (Liu et al., 2008; Xie et al., 2012; Ma et al., 2014a; Cai et al., 2015b; Zhao W. et al., 2015; Wang Z. et al., 2016). The present study elucidated overexpression of USF1 in GECs increased the expressions of ZO-1, occludin, and claudin-5 as well as decreased BTB permeability, and vice versa. The results of CHIP showed USF1 was, respectively, combined with the promoter regions of tight junction related proteins *ZO-1, occludin*, and *claudin-5* and increased their promoter activity. Our findings had proved that *ZO-1, occludin*, and *claudin-5* were the target genes of transcription factor USF1. Other studies were basically consistent with our findings about USF1 increasing promoter activity of target gene. USF1 was reported to be able to combine with E-box sequence in the promoter of cathepsin B and increase its promoter activity as well as expression, and accordingly regulate the invasion and development of tumor (Yan et al., 2003). In human vascular smooth muscle cells, USF1 not only bound to E-box sequence in the promoter of cGMP dependent protein kinase 1 but also increased its promoter activity and expression, and thus regulated the growth and differentiation of vascular smooth cell (Sellak et al., 2005). Besides, USF1 participated in the transcription of ~40 kinds of cardiovascular related genes (Kristiansson et al., 2008), whereas the regulatory effect of USF1 on vascular endothelial cells still needs more research.

Given all that, this study for the first time proved that HOTAIR, miR-148b-3p, and transcription factor USF1 were expressed in ECs and GECs, and clarified the target combination and binding sites between HOTAIR and miR-148b-3p as well as miR-148b-3p and USF1. Our findings also suggested that tight junction related proteins ZO-1, occludin, and claudin-5 were the target genes of transcription factor USF1 and further pointed out the probably mechanisms of HOTAIR/miR-148b-3p/USF1 in regulating BTB permeability. This reciprocal effect might provide new strategies for selective BTB opening and novel targets for glioma treatment.

## Author contributions

Study concept and design: YX and YHL. Acquisition of data: LS, YL, ZL, JM, and HC. Analysis and interpretation of data: LS, LZ, JM, HC, and ZL. Drafting of the manuscript: LS, YL, PW, and LZ. Critical revision of the manuscript for important intellectual content: YX, PW, LL, and LZ. Final approval of the version to be published: YX. Administrative, technical, and material support: YX, YHL, PW, and LL. Besides this they all agree to be accountable for all aspects of the work.

### Conflict of interest statement

The authors declare that the research was conducted in the absence of any commercial or financial relationships that could be construed as a potential conflict of interest.

## Abbreviations

lncRNAs: long non-coding RNAs
HOTAIR: homeobox transcript antisense intergenic RNA r
USF1: upstream stimulating factors1
3′UTR: 3′untranslated region
hCMEC/D3: human cerebral microvascular endothelial cell
ECs: endothelial cells
GECs: glioma microvascular endothelial cells
ZO-1: Zonula occluden-1
HRP: horseradish peroxidase
TEER: transendothelial electric resistance
IDVs: integrated density values
ChIP: chromatin immunoprecipitation
DAPI: diamidino phenylindole.
